# Mathematical Approach to Investigate Stress due to Control Measures to Curb COVID-19

**DOI:** 10.1155/2022/7772263

**Published:** 2022-01-13

**Authors:** James Nicodemus Paul, Silas Steven Mirau, Isambi Sailon Mbalawata

**Affiliations:** ^1^School of Computational and Communication Science and Engineering, The Nelson Mandela, African Institution of Science and Technology, P.O. Box 447, Arusha, Tanzania; ^2^African Institute for Mathematical Sciences, NEI Global Secretariat, rue KG590 St., Kigali, Rwanda

## Abstract

COVID-19 is a world pandemic that has affected and continues to affect the social lives of people. Due to its social and economic impact, different countries imposed preventive measures that are aimed at reducing the transmission of the disease. Such control measures include physical distancing, quarantine, hand-washing, travel and boarder restrictions, lockdown, and the use of hand sanitizers. Quarantine, out of the aforementioned control measures, is considered to be more stressful for people to manage. When people are stressed, their body immunity becomes weak, which leads to multiplying of coronavirus within the body. Therefore, a mathematical model consisting of six compartments, Susceptible-Exposed-Quarantine-Infectious-Hospitalized-Recovered (*SEQIHR*) was developed, aimed at showing the impact of stress on the transmission of COVID-19 disease. From the model formulated, the positivity, bounded region, existence, uniqueness of the solution, the model existence of free and endemic equilibrium points, and local and global stability were theoretically proved. The basic reproduction number (*R*_0_) was derived by using the next-generation matrix method, which shows that, when *R*_0_ < 1, the disease-free equilibrium is globally asymptotically stable whereas when *R*_0_ > 1 the endemic equilibrium is globally asymptotically stable. Moreover, the Partial Rank Correlation Coefficient (PRCC) method was used to study the correlation between model parameters and *R*_0_. Numerically, the *SEQIHR* model was solved by using the Rung-Kutta fourth-order method, while the least square method was used for parameter identifiability. Furthermore, graphical presentation revealed that when the mental health of an individual is good, the body immunity becomes strong and hence minimizes the infection. Conclusively, the control parameters have a significant impact in reducing the transmission of COVID-19.

## 1. Introduction

Coronavirus disease-2019 (COVID-19) is an infectious disease caused by a newly discovered coronavirus named severe acute respiratory syndrome coronavirus-2 (SARS-COV-2). This pandemic originated in Wuhan, China, with the first case reported in December 2019, and has spread to other parts of the world in early 2020 as discussed in [1, 2]. When the total confirmed cases globally were 125,260 and 4613 deaths in 24 hours, the World Health Organization (WHO), on 12th March 2020, announced COVID-19 disease as the World pandemic as presented in [3]. The global leaders were greatly bothered by this disease due to its fast spread from one person to another and its social and economic impact on their respective countries. The WHO and country leaders focused on finding ways to reduce the transmission of the disease by introducing some measures such as lockdown, quarantine, closing borders, travel bans, and isolation centers [4–7].

Mathematical models are essential tools in evaluating various transmission and control intervention programs for infectious diseases. There are a number of mathematical models on COVID-19 pandemic developed from the start of this human disturbing disease [8]. The author discusses social isolation measures taken by the government in Brazil to fight COVID-19 disease, and also, the protection of health workers was discussed by Masandawa et al. [9]. In their study, Khan et al. [10] discussed on isolation and quarantine as the best ways of fighting COVID-19 disease. At the beginning of the pandemic, many ways to fight the disease were introduced by many scientists. Ullah and Khan [11] explored several ways such as social distancing, self-isolation, quarantine, and hospitalization and concluded that these are the best ways to curb COVID-19. Dos Santos [12], in his review, studied on the effects of social distancing and social isolation measures as good ways to fight against the disease, although they lead to social stress which influences the spread of the disease. Early 2020, some mathematical models for COVID-19 were developed and published. Dhanwant and Ramanathan [13] explored how the social distancing in India during the pandemic helped to reduce the transmission of COVID-19 disease because the spread of the disease is by social contact. Khan and Atangana [14] discussed the interaction of bats and unknown hosts and then the interaction of people in the seafood market where there is enough source of infection. They presented their results graphically to show how they can minimize the infections.

Ashcroft et al. [15] discussed the impact of quarantine on the transmission of COVID-19 disease showing that many countries impose quarantine to ensure the exposed people and those from abroad are isolated for a specific period of time to prevent the spread of the disease. However, these measures took a larger economical toll and affected the health of the isolated individuals. Prati [16], from Italy, discussed the national impacts of quarantine psychologically. In their online survey of 1569 people living in Italy, they found that there are psychosocial factors that influence the disease, such as media exposure to COVID-19 outbreak, financial loss, higher worry, and negative attitude towards quarantine leading to psychological impacts. The mental health of public and healthcare professionals is affected by the pandemic, especially during quarantine time where hypervigilance arises because of fear and anxiety [17, 18].

Stress affects many quarantined people whereby their immune system is disturbed by the COVID-19, and this is most likely because during quarantine, people are isolated from their families and community members, so they develop fear, and later, the body becomes stressed which affects their immune system. When the immune system is disturbed, it fails to fight against the intruders, which leads to the fast spread of COVID-19 throughout the body. Therefore, this research is aimed at formulating a deterministic model to explore the impact of stress in quarantine to the human population. The model has six compartmental classes (Susceptible, Exposed, Quarantine, Infectious, Hospitalized, and Recovered). The model is extended from the model given in [19] by incorporating the hospitalized class and introducing a stress parameter in a quarantined and infected class.

The introduction of this work presented in Section 1. Model formulation, discussion of its compartments, and parameters are presented in Section 2.  Section 3 contains the discussion of the model analysis theoretically, which includes positivity and bounded regions, the existence, uniqueness of the model, reproduction number, and local and global stability of the COVID-19 disease.  Section 4 deals with a discussion of numerical simulation for the model, including sensitivity analysis, numerical solutions, PRCC results, parameter identifiability, and model fitting by the least square method are presented.  Section 5 concludes this work and contains the possible extension of this model.

## 2. Model Formulation

In this study, a mathematical model for COVID-19 was formulated based on realistic assumptions. The total population model *N*(*t*) is divided into six human subclasses, namely, susceptible *S*(*t*) (those who are at risk to contact COVID-19 infection), exposed *E*(*t*) (the population which is infected but not infectious), quarantined *Q*(*t*) (those who contacted a COVID-19-infected individual but did not develop any symptom), infectious *I*(*t*) (those who have COVID-19 symptoms and are capable of spreading the disease), hospitalized *H*(*t*) (infectious individuals admitted to a healthcare facility (active cases)), and recovered *R*(*t*) (those recovered from the COVID-19).

### 2.1. Model Assumptions

By presenting an infectious disease with a mathematical model, the following assumptions for the *SEQIHR* model are considered based on the characteristics of COVID-19 disease in this work.

- All members of the population can have an equal chance of getting a COVID-19 disease
- Stress in a quarantined class is higher than that in an infectious class
- Population from outside the country were taken directly to quarantine class
- All compartments have an equal natural death rate
- The death due to the disease may be only in two variables (infectious and hospitalized)
- Recruitment rates (Newborns) are assumed to be susceptible
- Individuals are equally likely to be infectious to the infected individuals when coming into contact
- Infected individuals are identified early and isolated (hospitalized) immediately for treatment
- There are only two options, a patient will either recover or die, which means no treatment failure
- The population differs within a given time step where recruitment and leaving rates differ

### 2.2. Model Compartments and Dynamics

From Section 2.1, the variable and parameter descriptions are to be presented by the following *SEQIHR* model compartmental diagram:

Let *N* be the total population divided; the transmission dynamics of COVID-19 disease in a population are shown in Figure 1. Consider Table 1, showing the variables and their descriptions:

The total population *N*(*t*) is given by the mathematical equation:

(1) $$\begin{array}{c} N\left(t\right)=S\left(t\right)+Q\left(t\right)+E\left(t\right)+I\left(t\right)+H\left(t\right)+R\left(t\right), \end{array}$$

where *t* ∈ [0, *t*] and *t* > 0.

Table 2 shows the model parameters and their descriptions:

The model parameters found in Equation (2) are described in Table 2. By considering the *SEQIHR* model with six compartments in Figure 1, the following are the transmission phases:

The Susceptible class, *S*(*t*), increases by the addition of a recruitment rate, *μ*. It also decreases by infection, if contacted with an infected individual at the rate of *β* and natural death at the rate of *b*.

An individual enters the Exposed class, *E*(*t*), after direct contact with an infected person, with an infection rate *β*. Furthermore, taking to hospital decreases the rate of *ω* and *q* for individuals with multiple symptoms. Individuals with clear (direct) symptoms are presented by (1-*ω*), and those with no symptoms are represented by *θ*, and then, the population in *E*(*t*) class is diminished by a leaving rate of natural death *b*.

The Quarantined class, *Q*(*t*), was formed by individuals' progress from exposed, *θ*, and population rate from outside the country, *ϕ*, also decreased by individuals with no symptoms after being tested. Then, the individuals with no infections going back to the susceptible class are presented by *α* and those infected individuals after being tested, going to the infectious class at the rate of *η*_1_ and diminishing by leaving a natural death rate of *b*.

The Infectious class, *I*(*t*), are individuals who progress from exposed at the rate of (1-*ω*) and then quarantine at the rate of *η*_1_. Additionally, this class decreases with hospitalized individuals at the rate of *η*_2_ and recovered at the rate of *ν*. Not only that but also it diminished by leaving the rate of natural death, *b*, and death due to the disease, *δ*.

The Hospitalized class, *H*(*t*), are individuals who progress from the exposed class at the rate of *ω* and *q*, then from the infectious compartment at the rate of *η*_2_. Individuals recovered from hospitalized class at the rate of *λ* and diminished by leaving the rate of natural death, *b*, and death due to COVID-19 disease, *δ*.

The Recovered class, *R*(*t*), are individuals who progress from a hospitalized compartment at the rate of *λ* and infectious rate *ν* and decrease by recovered individuals who are going back to the susceptible population *ρ* and then diminished by the leaving rate of *b*.

### 2.3. Model Equations

Based on the assumptions made and the relationship that exists between the variables shown in Figure 1, the system of six ordinary differential equations is formed as in

(2) $$\begin{array}{c} \frac{dS}{dt}=\mu +\alpha Q+\rho R-\beta IS-bS, \end{array}$$

(3) $$\begin{array}{c} \frac{dE}{dt}=\beta IS-\theta E-qE-bE, \end{array}$$

(4) $$\begin{array}{c} \frac{dQ}{dt}=\phi +\theta E-\alpha Q-\eta_{1}Q-bQ, \end{array}$$

(5) $$\begin{array}{c} \frac{dI}{dt}=\left(1-\omega \right)qE+\eta_{1}Q-\eta_{2}I-\nu I-\delta I-bI, \end{array}$$

(6) $$\begin{array}{c} \frac{dH}{dt}=\omega qE+\eta_{2}I-\lambda H-\delta H-bH, \end{array}$$

(7) $$\begin{array}{c} \frac{dR}{dt}=\lambda H+\nu I-\rho R-bR. \end{array}$$

## 3. Model Analysis

In this section, positivity, boundedness, derived equilibrium states, basic reproduction number, and stability analysis are discussed.

### 3.1. Positivity of the Model

For the model equations to be epidemiologically, we need to prove that the state variables are nonnegative ∀*t* ≥ 0.

**Theorem 1 .**

Let the initial data set be (*S*, *E*, *Q*, *I*, *H*, *R*)(0) > 0. The solution set of the model system 2 is positive ∀*t* > 0.

**Proof**

From the system of model Equation (2), consider the first equation:

(8) $$\begin{array}{c} \frac{dS}{dt}=\mu +\alpha Q+\rho R-\left(\beta I+b\right)S. \end{array}$$

By considering the negative term, by ignoring the rest, Equation (8) is reduced to

(9) $$\begin{array}{c} \frac{dS}{dt}\geq -\left(\beta I+b\right)S. \end{array}$$

This is the first-order linear differential inequality which can be solved by a separable method *y*′ = *f*(*x*)*g*(*y*) (where *S* ≥ 0) resulting in

(10) $$\begin{array}{c} \int_{S\left(0\right)}^{S\left(t\right)}\frac{dS}{S}\geq -\int_{0}^{t}\left(\beta I+b\right)dt,S\left(t\right)\geq S\left(0\right)e^{-\left(\beta I+b\right)t}, \end{array}$$

in the absence of COVID-19 disease,

(11) $$\begin{array}{c} S\left(t\right)\geq S\left(0\right)e^{-bt},\;S\left(0\right)\geq 0,\forall t>0. \end{array}$$

By applying the same procedure to the remaining equations, the results are *E*(0) ≥ 0, *Q*(0) ≥ 0, *I*(0) ≥ 0, *H*(0) ≥ 0, and *R*(0) ≥ 0. Therefore, the set of solutions *S*(*t*), *E*(*t*), *Q*(*t*), *I*(*t*), *H*(*t*), and *R*(*t*) of the model is positive ∀*t* > 0.

### 3.2. Invariant (Boundedness) Region

The *SEQIHR* model is represented by differential equations in system 2, which is to be analyzed in a feasible region *Ω*, and all state variables and parameters of the model are assumed to be positive ∀*t* ≥ 0. The bounded region is obtained through the following theorem.

**Theorem 2 .**

The set *Ω* is positively invariant and attracts all solutions in ℝ_+_^6^.

**Proof**

Since *N*(*t*) = *S*(*t*) + *Q*(*t*) + *E*(*t*) + *I*(*t*) + *H*(*t*) + *R*(*t*), then the derivative of *N*(*t*) is given as

(12) $$\begin{array}{c} \frac{dN}{dt}=\frac{dS}{dt}+\frac{dE}{dt}+\frac{dQ}{dt}+\frac{dI}{dt}+\frac{dH}{dt}+\frac{dR}{dt}. \end{array}$$

Substituting model Equation (2) to Equation (12) gives

(13) $$\begin{array}{c} \frac{dN}{dt}=\left\{\begin{array}{c} \left(\mu +\alpha Q+\rho R-\beta IS-bS\right)+\left(\beta IS-\theta E-qE-bE\right)\\ +\left(\phi +\theta E-\alpha Q-\eta_{1}Q-bQ\right)+\left(\left(1-\omega \right)qE+\eta_{1}Q-\eta_{2}I-\nu I-\delta I-bI\right)\\ +\left(\omega qE+\eta_{2}I-\lambda H-\delta H-bH\right)+\left(\lambda H+\nu I-\rho R-bR\right). \end{array}\right. \end{array}$$

Further simplification leads to

(14) $$\begin{array}{c} \frac{dN}{dt}=\mu +\phi -\left(S+E+Q+I+H+R\right)b-\left(\delta I+\delta R\right), \end{array}$$

implying that

(15) $$\begin{array}{c} \frac{dN}{dt}=\mu +\phi -Nb-\left(\delta I+\delta R\right). \end{array}$$

For disease-free, *δI*⟹0 and *δR*⟹0, then (*dN*/*dt*) ≤ *μ* + *ϕ* − *Nb*.

This is a first-order linear differential equation, by a separable method.

(16) $$\begin{array}{c} \int_{N\left(0\right)}^{N\left(t\right)}\frac{dN}{\left(\mu +\phi -bN\right)}\leq \int_{0}^{t}dt,⟹N\left(t\right)\geq \frac{\mu +\phi }{b}\left(1-e^{-bt}\right)+N\left(0\right)e^{-bt}. \end{array}$$

When *t* = 0, *N*(0) ≥ 0. When *t*⟹∞ then, *N*(∞) ≤ (*μ* + *ϕ*)/*b*.

The Invariant region is given by *Ω* = (*S*, *E*, *Q*, *I*, *H*, *R*) ∈ ℝ_+_^6^ : 0 ≤ *N*(*t*) ≤ (*μ* + *ϕ*)/*b*. The *SEQIHR* model is biologically and epidemiologically meaningful; thus, we can consider the flow generated by the model for analysis.

### 3.3. Existence and Uniqueness of the Solution

From the first-order differential equation given in the form: *y*′ = *f*(*t*, *y*), *y*(*t*_0_) = *y*_0_. The following questions will be of interest:

- Under what conditions can we say that a solution to the equation *y*′ exists?
- Under what conditions does a unique solution exist to the equation *y*′?

Consider the following equations to answer the question.

(17) $$\begin{array}{c} f_{1}=\mu +\alpha Q+\delta R-\beta IS-bS, \end{array}$$

(18) $$\begin{array}{c} f_{2}=\beta IS-\theta E-qE-bE, \end{array}$$

(19) $$\begin{array}{c} f_{3}=\phi +\theta E-\left(\alpha +\eta_{1}+b\right)Q, \end{array}$$

(20) $$\begin{array}{c} f_{4}=\left(1-\omega \right)qE+\eta_{1}Q-\left(\eta_{2}+\nu +\delta +b\right)I, \end{array}$$

(21) $$\begin{array}{c} f_{5}=\omega qE+\eta_{2}I-\left(\lambda +\delta +b\right)H, \end{array}$$

(22) $$\begin{array}{c} f_{6}=\lambda H+\nu I-\left(\rho +b\right)R. \end{array}$$

#### 3.3.1. Uniqueness of Solution

**Theorem 3 .**

Let us use *D* to denote the domain:

(23) $$\begin{array}{c} \left|t-t_{0}\right|\leq a,\left\|y-y_{0}\right\|\leq b,y=\left(y_{1},y_{2},\cdots ,y_{n}\right),\;y_{0}=\left(y_{1}0,y_{2}0,\cdots ,y_{n}0\right). \end{array}$$

**Proof**

Suppose *f*(*t*, *y*) satisfies the Lipschitz condition; therefore,

(24) $$\begin{array}{c} \left\|f\left(t,y_{2}\right)\right\|-\left\|f\left(t,y_{1}\right)\right\|\leq k\left\|x_{2}-x_{1}\right\|. \end{array}$$

Whenever the points (*t*, *x*_1_) and (*t*, *x*_2_) belong to the domain D and *k* is used to represent the positive constant, then, there exist a constant *α* > 0 and a unique solution *y*(*t*) of system 11 in the interval |*t* − *t*_0_| ≤ *α*. It is essential to note that condition (24) is satisfied by (*∂f*_*i*_/*∂y*_*j*_), *i*, *j* = 1, 2, 3, ⋯, *n* to be continuous and bounded in domain D.

If *f*(*t*, *y*) has a continuous partial derivative (*∂f*_*i*_/*∂y*_*j*_) on a bounded closed convex domain ℝ (i.e., the convex set of real numbers), where ℝ is used to denote real numbers; then it satisfies a Lipschitz condition in ℝ. Our interest is in the domain:

(25) $$\begin{array}{c} 1\leq \varepsilon \leq \mathbb{R}. \end{array}$$

Therefore, we look for the bounded solution of the form 0 < ℝ < ∞.

#### 3.3.2. Existence of a Solution

**Theorem 4 .**

Let the domain be denoted by *D*, also defined in Equation (23), such that Equations (24) and (25) hold. Then, the existing solution of Equation (2) is bounded in the domain *D*.

**Proof**

From Equations (10)–(15), by showing that $\left\{\begin{array}{c} \left(\partial f_{i}/\partial y_{j}\right),i,j=1,2,3,4,5,6, \end{array}\right.$ then, Equations (1) and (2) are continuous and bounded. That means the partial derivatives are continuous and bound. Consider the exploration of the partial derivatives for all model equations.

From Equation (17), we obtain the following system of equations:

(26) $$\begin{array}{c} \frac{\partial f_{1}}{\partial S}=-\beta I-b,\left|\frac{\partial f_{1}}{\partial S}\right|=\left|-\beta I-b\right|<\infty ,\\ \frac{\partial f_{1}}{\partial E}=0,\left|\frac{\partial f_{1}}{\partial E}\right|=\left|0\right|<\infty ,\\ \frac{\partial f_{1}}{\partial Q}=\alpha ,\left|\frac{\partial f_{1}}{\partial Q}\right|=\left|\alpha \right|<\infty ,\\ \frac{\partial f_{1}}{\partial I}=-\beta S,\left|\frac{\partial f_{1}}{\partial I}\right|=\left|-\beta S\right|<\infty ,\\ \frac{\partial f_{1}}{\partial H}=0,\left|\frac{\partial f_{1}}{\partial H}\right|=\left|0\right|<\infty ,\\ \frac{\partial f_{1}}{\partial R}=\rho ,\left|\frac{\partial f_{1}}{\partial R}\right|=\left|\rho \right|<\infty . \end{array}$$

Similarly, from Equation (18), we obtain the following system of equations:

(27) $$\begin{array}{c} \begin{array}{c} \begin{array}{c} \begin{array}{c} \frac{\partial f_{2}}{\partial S}=\beta I,\left|\frac{\partial f_{2}}{\partial S}\right|=\left|\beta I\right|<\infty ,\\ \frac{\partial f_{2}}{\partial E}=-\left(\theta +q+b\right),\left|\frac{\partial f_{2}}{\partial E}\right|=\left|-\left(\theta +q+b\right)\right|<\infty , \end{array}\\ \frac{\partial f_{2}}{\partial Q}=0,\left|\frac{\delta f_{2}}{\partial Q}\right|=\left|0\right|<\infty ,\\ \frac{\partial f_{2}}{\partial I}=\beta S,\left|\frac{\partial f_{2}}{\partial I}\right|=\left|\beta S\right|<\infty , \end{array}\\ \frac{\partial f_{2}}{\partial H}=0,\left|\frac{\partial f_{2}}{\partial H}\right|=\left|0\right|<\infty ,\\ \frac{\partial f_{2}}{\partial R}=0,\left|\frac{\partial f_{2}}{\partial R}\right|=\left|0\right|<\infty . \end{array} \end{array}$$

The same procedures are taken for Equations (19), (20), (21), and (22). Therefore, all partial derivatives are continuous and bounded; hence, from Theorem 4, it is concluded that there exists a unique solution of the model in Equation (2) in the domain region *D*.

### 3.4. Existence of Disease-Free Equilibrium Point (DFE)

The disease-free equilibrium point, obtained when the infected components are zero, can be done by setting the right-hand side of the equation equal to zero, as in

(28) $$\begin{array}{c} \frac{dS}{dt}=\frac{dE}{dt}=\frac{dQ}{dt}=\frac{dI}{dt}=\frac{dH}{dt}=\frac{dR}{dt}=0. \end{array}$$

When there is no disease, then, *E*=0, *Q*=0, *I*=0, *H*=0, and *R*=0.

By considering each model equation from Equation (2),

(29) $$\begin{array}{c} \mu +\alpha Q+\rho R-\beta IS-bS=0\text{ gives }\mu -bS=0,\text{ then},\;S=\frac{\mu }{b}. \end{array}$$

In addition to the second model equation,

(30) $$\begin{array}{c} \begin{array}{c} \beta IS=\left(\theta +q+b\right)E=0\text{ gives }E=\frac{\beta IS}{\theta +q+b},\text{ but }\beta =0,\text{ then},\;E=0. \end{array} \end{array}$$

Similarly, for the third model equation,

(31) $$\begin{array}{c} \begin{array}{c} \phi +\theta E-\alpha Q-\eta_{1}Q-bQ=0\text{ gives }Q=\frac{\phi +\theta E}{\alpha +\eta_{1}+b},\text{but},E=0, \end{array} \end{array}$$

then,

(32) $$\begin{array}{c} Q=\frac{\phi }{\alpha +\eta_{1}+b}. \end{array}$$

By considering the same procedures for the fourth, fifth, and sixth model equations, the following is obtained:

(33) $$\begin{array}{c} I=0,H=0,R=0. \end{array}$$

Therefore,

(34) $$\begin{array}{c} E_{0}=\left(S^{0},E^{0},Q^{0},I^{0},H^{0},R^{0}\right)={\left(\frac{\mu }{b},0,\frac{\phi }{\alpha +\eta_{1}+b},0,0,0\right)}^{T}. \end{array}$$

Equation (34) represents the state in which there is no infection and is known as the disease-free equilibrium point.

### 3.5. Basic Reproduction Number (*R*_0_)

The basic reproduction number *R*_0_ is the midpoint number of infections caused by an infectious individual during the entire period of infectiousness [20]. In an epidemiology study, the basic reproduction number is a nondimensional quantity that sets the threshold during the study, both for predicting the outbreak and for evaluating the control strategies. Additionally, *R*_0_ analyzes the equilibrium stability, *R*_0_ < 1, which means that infectious individuals will cause less than one secondary infection and die out. Every infectious individual infects more than one secondary infection when *R*_0_ > 1, and the disease spreads to the population. In the *SEQIHR* model, the basic reproduction number is computed by using the next-generation matrix approach [21] and then obtained by taking the dominant eigenvalues (Spectral radius). Let *F*_*i*_(*x*) be the rate of new infection in compartment *i* and *V*_*i*_ be the rate of transfer of individuals into compartment *i* by all means other than the epidemic. The important thing is to obtain the disease-free equilibrium point *E*_0_. Thus, the computed matrices F and V which are *n* × *n* matrices, where *n* represents the infected classes, defined by: *F* = ((*∂F*_*i*_/*∂x*_*j*_)(*E*_0_)) and *V* = ((*∂V*_*i*_/*∂x*_*j*_)(*E*_0_)), where 1 ≤ *i*, *j* ≤ *n*, *F* are nonnegative, and *V* is a nonsingular *n*-matrix (the matrix with inverse belongs to the class of positive matrices). Since *F* is nonnegative and *V* is a nonsingular matrix, then *V*^−1^ and *FV*^−1^ are nonnegative. Therefore, the next-generation matrix *FV*^−1^ is computed as defined by [22].

Note that the basic reproduction number is defined as the spectral radius (dominant eigenvalue) of the matrix *FV*^−1^ [23], that is,

(35) $$\begin{array}{c} R_{0}=\rho \left(FV^{-1}\right),\\ FV^{-1}=\left[\frac{\partial F_{i}}{\partial x_{j}}\left(E_{0}\right)\right]{\left[\frac{\partial V_{i}}{\partial x_{j}}\left(E_{0}\right)\right]}^{-1}. \end{array}$$

where *F* is the rate of new infection in compartment *I*. The new forces of infection are

(36) $$\begin{array}{c} \begin{array}{c} \begin{array}{c} \frac{dE}{dt}=\beta IS-\left(\theta +q+b\right)E,\\ \frac{dQ}{dt}=\phi +\theta E-\left(\alpha +\eta_{1}+b\right)Q, \end{array}\\ \frac{dI}{dt}=\left(1-\omega \right)qE+\eta_{1}Q-\left(\eta_{2}+\nu +\delta +b\right)I,\\ \frac{dH}{dt}=\omega qE+\eta_{2}I-\left(\lambda +\delta +b\right)H. \end{array} \end{array}$$

From Equation (36), when *I* and *S* meet, we obtain the following:

(37) $$\begin{array}{c} F_{i}=\left(\begin{array}{c} f_{1}\\ f_{2}\\ f_{3}\\ f_{4} \end{array}\right)=\left(\begin{array}{c} \beta IS\\ 0\\ 0\\ 0 \end{array}\right), \end{array}$$

From Equation (37), the Jacobian matrix of disease-free equilibrium (DFE) is given by

(38) $$\begin{array}{c} F_{J}=\left(\begin{array}{cccc} 0 & 0 & \beta S & 0\\ 0 & 0 & 0 & 0\\ 0 & 0 & 0 & 0\\ 0 & 0 & 0 & 0 \end{array}\right). \end{array}$$

The partial derivative of Equation (38) with respect to *E*, *Q*, *I*, and *H* is given as

(39) $$\begin{array}{c} V=\left(\begin{array}{cccc} b+\theta +q & 0 & 0 & 0\\ -\theta & \alpha +b+\eta_{1} & 0 & 0\\ \left(\omega -1\right)q & -\eta_{1} & b+\delta +\eta_{2}+v & 0\\ -\omega & 0 & -\eta_{2} & b+\delta +\lambda \end{array}\right), \end{array}$$

Given that *A*_1_ = *b* + *α* + *η*_1_ and *A*_2_ = *b* + *δ*+*η*_2_ + *ν*. The inverse of *V* is

(40) $$\begin{array}{c} V^{-1}=\left(\begin{array}{cccc} \frac{1}{b+\theta +q} & 0 & 0 & 0\\ \frac{\theta }{A_{1}\left(b+\theta +q\right)} & \frac{1}{A_{1}} & 0 & 0\\ \frac{-\alpha \omega +\alpha +b\left(-\omega \right)+b+\eta_{1}\theta -\eta_{1}\omega +\eta_{1}}{A_{1}A_{2}\left(b+\theta +q\right)} & \frac{\eta_{1}}{A_{1}A_{2}} & \frac{1}{A_{2}} & 0\\ \frac{A_{1}A_{2}\omega +\eta_{2}\left(-\alpha \omega +\alpha +b\left(-\omega \right)+b+\eta_{1}\theta -\eta_{1}\omega +\eta_{1}\right)}{A_{1}A_{2}\left(b+\delta +\lambda \right)\left(b+\theta +q\right)} & \frac{\eta_{1}\eta_{2}}{A_{1}A_{2}\left(b+\delta +\lambda \right)} & \frac{\eta_{2}}{A_{2}\left(b+\delta +\lambda \right)} & \frac{1}{b+\delta +\lambda } \end{array}\right). \end{array}$$

The product matrix *FV*^−1^ is given by:

(41) $$\begin{array}{c} FV^{-1}=\left(\begin{array}{cccc} \frac{\beta \mu \left(\eta_{1}\theta -q\left(\omega -1\right)\left(\alpha +b+\eta_{1}\right)\right)}{b\left(\alpha +b+\eta_{1}\right)\left(b+\theta +q\right)\left(b+\delta +\eta_{2}+\nu \right)} & \frac{\beta \eta_{1}\mu }{b\left(\alpha +b+\eta_{1}\right)\left(b+\delta +\eta_{2}+\nu \right)} & \frac{\beta \mu }{b\left(b+\delta +\eta_{2}+\nu \right)} & 0\\ 0 & 0 & 0 & 0\\ 0 & 0 & 0 & 0\\ 0 & 0 & 0 & 0 \end{array}\right),\\ \text{Eigenvalues}\;=\left\{0,0,0,\frac{\beta \mu \left(-bq\omega +bq+\eta_{1}\theta -\alpha q\omega +\alpha q-\eta_{1}q\omega +\eta_{1}q\right)}{b\left(\alpha +b+\eta_{1}\right)\left(b+\theta +q\right)\left(b+\delta +\eta_{2}+\nu \right)}\right\},\\ \lambda_{1}=0,\lambda_{2}=0,\lambda_{3}=0,\lambda_{4}=\frac{\beta \mu \left(\eta_{1}\left(\theta +q\left(-\omega \right)+q\right)-q\left(\omega -1\right)\left(\alpha +b\right)\right)}{b\left(\alpha +b+\eta_{1}\right)\left(b+\theta +q\right)\left(b+\delta +\eta_{2}+\nu \right)}. \end{array}$$

Thus, the basic reproduction number becomes

(42) $$\begin{array}{c} R_{0}=\frac{\beta \mu \left(\eta_{1}\left(\theta -\omega q+q\right)+q\left(1-\omega \right)\left(\alpha +b\right)\right)}{b\left(\alpha +b+\eta_{1}\right)\left(b+\theta +q\right)\left(b+\delta +\eta_{2}+\nu \right)}. \end{array}$$

### 3.6. Existence of Endemic Equilibrium Point

Endemic equilibrium points are the steady-state solutions whereby the disease persists in the population [24]. The stability analysis of the endemic equilibrium point describes the long-term dynamics of COVID-19 in the population [25]. By solving all systems of differential equations from the model Equation (2), all derivatives are equal to zero (solve for all variables simultaneously).

**Theorem 5 .**

The endemic equilibrium point of model Equation (2) is locally asymptotically stable in the region *Ω* if *R*_0_ < 1 and unstable if *R*_0_ > 1.

**Proof**

At the endemic equilibrium point *S* = *S*^∗^, *E* = *E*^∗^, *Q* = *Q*^∗^, *I* = *I*^∗^, *H* = *H*^∗^, and *R* = *R*^∗^. The variables are given as follows:

(43) $$\begin{array}{c} S^{*}=\frac{\mu +\alpha Q+\rho R}{b+\beta I}E^{*}=\frac{\beta IS}{b+\theta +q}Q^{*}=\frac{\phi +\theta E}{b+\alpha +\eta_{1}}H^{*}=\frac{E\omega q+\eta_{2}I}{b+\delta +\lambda }R^{*}=\frac{H\lambda +\nu I}{b+\rho },\\ I^{*}=\frac{\mu \left(\phi \eta_{1}+A_{1}A_{2}\left(R_{0}-1\right)\right)+R_{0}\left(\alpha Q^{*}+\rho R^{*}\right)A_{1}A_{2}}{\beta \mu \left(A_{1}A_{2}-\phi \eta_{1}\right)}. \end{array}$$

### 3.7. Local Stability of the Disease-Free Equilibrium

The eigenvalues, which are determined by finding the partial derivatives of the vector-valued function, are used to study the local stability of the disease-free equilibrium. If the Jacobian matrix evaluated at that point has negative eigenvalues, the equilibrium point is asymptotically stable. The Routh-Hurwitz criterion in [26] will be utilized to demonstrate the local stability in this work.

**Theorem 6 .**

The disease-free equilibrium point *E*_0_ is locally asymptotically stable if *R*_0_ < 1, and it is unstable when *R*_0_ > 1.

**Proof**

The linearization of the system of model 2 is done by computing its Jacobian matrix to prove this theorem. At the disease-free equilibrium point, the partial derivatives of each equation in the system for state variables *S*, *E*, *Q*, *I*, *H*, *R*, which are used to generate the Jacobian matrix *J*_*E*_0__ as in 21.

(44) $$\begin{array}{c} J_{E_{0}}=\left(\begin{array}{cccccc} -b & 0 & \alpha & -\beta \text{S} & 0 & \rho \\ 0 & -b-\theta -q & 0 & \beta \text{S} & 0 & 0\\ 0 & \theta & -\alpha -b-\eta_{1} & 0 & 0 & 0\\ 0 & q\left(1-\omega \right) & \eta_{1} & -b-\delta -\eta_{2}-\nu & 0 & 0\\ 0 & \omega \text{q} & 0 & \eta_{2} & -b-\delta -\lambda & 0\\ 0 & 0 & 0 & \nu & \lambda & -b-\rho \end{array}\right). \end{array}$$

At a disease-free equilibrium,

(45) $$\begin{array}{c} S=\frac{\mu }{b},I=0. \end{array}$$

The disease-free equilibrium will be asymptotically stable if the eigenvalues of *J*_*E*_0__ < 0.

(46) $$\begin{array}{c} \left|\begin{array}{cccccc} -b & 0 & \alpha & -\frac{\beta \mu }{b} & 0 & \rho \\ 0 & -b-\theta -q & 0 & \frac{\beta \mu }{b} & 0 & 0\\ 0 & \theta & -\alpha -b-\eta_{1} & 0 & 0 & 0\\ 0 & q\left(1-\omega \right) & \eta_{1} & -b-\delta -\eta_{2}-\nu & 0 & 0\\ 0 & \omega \text{q} & 0 & \eta_{2} & -b-\delta -\lambda & 0\\ 0 & 0 & 0 & \nu & \lambda & -b-\rho \end{array}\right|=0. \end{array}$$

From matrix (46), it is clear that the first, second, and third eigenvalues are

(47) $$\begin{array}{c} \lambda_{1}=-b,\lambda_{2}=-b-\rho ,\text{and }\lambda_{3}=-b-\delta -\lambda . \end{array}$$

Then matrix (46) reduces to a 3 × 3 matrix after the cancellation of the respective rows and columns used to obtain the first, second, and third eigenvalues as shown in

(48) $$\begin{array}{c} J_{E_{0}}=\left(\begin{array}{ccc} -b-\theta -q & 0 & \frac{\beta \mu }{b}\\ \theta & -\alpha -b-\eta_{1} & 0\\ q\left(1-\omega \right) & \eta_{1} & -b-\delta -\eta_{2}-\nu \end{array}\right). \end{array}$$

The characteristic polynomial of matrix (48) is given in the form

(49) $$\begin{array}{c} Z\left(\lambda \right)=\lambda^{3}+a_{1}\lambda^{2}+a_{2}\lambda +a_{3}, \end{array}$$

where

(50) $$\begin{array}{c} a_{1}=\alpha +3b+\delta +\eta_{1}+\eta_{2}+\theta +\nu +q,\\ a_{2}=\alpha \delta +\alpha \eta_{2}+\alpha \theta +\alpha \nu +3b^{2}+2\alpha b+2b\delta +2b\eta_{1}+2b\eta_{2}+2b\theta +2b\nu -\frac{\beta \mu q}{b}+2bq+\delta \eta_{1}+\delta \theta +\eta_{1}\theta +\eta_{2}\theta +\eta_{1}\nu +\eta_{1}\eta_{2}+\theta \nu +\alpha q+\delta q+\eta_{1}q+\eta_{2}q+\nu q,\\ a_{3}=\alpha \delta \theta +\alpha \eta_{2}\theta +\alpha \theta \nu +b^{3}+\alpha b^{2}+b^{2}\delta +b^{2}\eta_{1}+b^{2}\eta_{2}+b^{2}\theta +b^{2}\nu +b^{2}q+\alpha b\delta +\alpha b\eta_{2}+\alpha b\theta +\alpha b\nu -\frac{\beta \eta_{1}\theta \mu }{b}+b\delta \eta_{1}+b\delta \theta +b\eta_{1}\theta +b\eta_{2}\theta +b\eta_{1}\nu +b\eta_{1}\eta_{2}+b\theta \nu +\frac{\alpha \beta \mu q\omega }{b}-\frac{\alpha \beta \mu q}{b}+\alpha bq+\frac{\beta \eta_{1}\mu q\omega }{b}-\frac{\beta \eta_{1}\mu q}{b}+b\delta q+b\eta_{1}q+b\eta_{2}q+b\nu q+\delta \eta_{1}\theta +\eta_{1}\theta \nu +\eta_{1}\eta_{2}\theta +\alpha \delta q+\alpha \eta_{2}q+\alpha \nu q+\beta \mu q\omega -\beta \mu q+\delta \eta_{1}q+\eta_{1}\nu q+\eta_{1}\eta_{2}q. \end{array}$$

However, *a*_1_ > 0, *a*_2_ > 0, and *a*_3_ > 0, condition *a*_1_*a*_2_ − *a*_3_ > 0.

(51) $$\begin{array}{c} a_{1}a_{2}-a_{3}=\frac{-\beta \mu q\omega \left(\alpha +b\right)+M_{1}\left(M_{2}-\beta \mu q\right)+M_{3}+\eta_{2}\left(M_{4}+M_{5}-\beta \mu q\right)+\eta_{1}\left(M_{6}+M_{7}+\beta \mu \left(\theta -q\omega \right)\right)}{b},\\ \frac{M_{1}M_{2}+M_{3}+\eta_{2}\left(M_{4}+M_{5}\right)+\eta_{1}\left(\beta \theta \mu +M_{6}+M_{7}\right)}{b}>\frac{\beta \mu q\omega \left(\alpha +b\right)+\beta \mu \eta_{2}q+\beta \mu M_{1}q+\mu q\omega \beta }{b}, \end{array}$$

where

(52) $$\begin{array}{c} M_{1}=2b+\delta +\theta +\nu +q,\\ M_{2}=4b^{3}+2b^{2}\left(2\alpha +\delta +\theta +\nu +q\right)+b\left(\alpha +\delta +\nu \right)\left(\alpha +\theta +q\right),\\ M_{3}=b\eta_{1}^{2}\left(2b+\delta +\eta_{2}+\theta +\nu +q\right),\\ M_{4}=8b^{3}+b\left(\alpha +\theta +q\right)\left(\alpha +2\delta +\theta +2\nu +q\right),\\ M_{5}=b^{2}\left(6\alpha +4\delta +6\theta +4\nu +6q\right)+b\eta_{2}\left(\alpha +2b+\theta +q\right),\\ M_{6}=8b^{3}+b^{2}\left(4\alpha +6\left(\delta +\theta +\nu \right)+6q\right)+b\left(\delta +\theta +\nu +q\right)\left(2\alpha +\delta +\theta +\nu +q\right),\\ M_{7}=b\eta_{2}\left(2\right.\left(\alpha +3b+\delta +\theta +\nu +q\right)+\eta_{2}. \end{array}$$

Hence, the condition *a*_1_*a*_2_ − *a*_3_ > 0 is satisfied. The Routh-Hurwitz criterion states that all elements of a system's characteristic polynomial must be negative in order for the system to be stable [27]. The disease is asymptotically stable because the eigenvalues are negative, and the Routh-Hurwitz requirements are satisfied.

### 3.8. Global Stability of Disease-Free Equilibrium Point (DFE)

The global stability of the *SEQIHR* model around the DFE will be proved. The stability result of DFE in epidemiological implication is that minimizing the COVID-19 infection cases will not generate an infection if *R*_0_ < 1.  Theorem 7 is considered.

**Theorem 7 .**

The DFE is globally asymptotically stable if *R*_0_ < 1, and unstable if *R*_0_ > 1.

**Proof**

Using the technique described in [23, 28], the studies examine the global stability of the model 1 disease-free equilibrium point. The format can be used to write the *SEQIHR* model as in

(53) $$\begin{array}{c} \left\{\begin{array}{c} \frac{dX_{n}}{dt}=A\left(X_{n}-X_{d_{f_{e}}}\right)+A_{1}X_{i},\\ \frac{dX_{i}}{dt}=A_{2}X_{i}. \end{array}\right. \end{array}$$

By considering Equation (54), *X*_*n*_ is the vector of the nontransmitting compartment, *X*_*i*_ is the vector of transmitting compartment, and *X*_*d*_*f*_*e*___ is the vector of disease-free equilibrium point.

(54) $$\begin{array}{c} X_{n}={\left(S,R\right)}^{T},X_{i}={\left(E,Q,I,H\right)}^{T},X_{d_{f_{e}}}=\left(\frac{1}{b},0\right), \end{array}$$

(55) $$\begin{array}{c} X_{n}-X_{d_{f_{e}}}=\left(\begin{array}{c} S-\frac{1}{b}\\ R \end{array}\right). \end{array}$$

We must show that the matrix *A* has real negative eigenvalues and *A*_2_ is a Metzler matrix in order for DFE to be globally stable (i.e., the off-diagonal elements of *A*_2_ are nonnegative, symbolically denoted by *A*_2_(*X*_*ij*_) ≥ ∀≠*j*). We can derive equations with and without transmission from model 1, as stated herewith.

(56) $$\begin{array}{c} \left(\begin{array}{c} \mu +\alpha Q+\rho R-\beta IS-bS\\ \lambda H+\nu I-\rho R-bR \end{array}\right)=A\left(\begin{array}{c} S-\frac{1}{b}\\ R \end{array}\right)+A_{1}\left(\begin{array}{c} \begin{array}{c} E\\ Q \end{array}\\ I\\ H \end{array}\right), \end{array}$$

(57) $$\begin{array}{c} \text{then},A=\left(\begin{array}{cc} -b & 0\\ 0 & -b \end{array}\right). \end{array}$$

The eigenvalues of the matrix *A* are located at the diagonal (-b and -b), and these eigenvalues are real, distinct, and negative. Moreover, matrices *A*_1_ and *A*_2_ are given by

(58) $$\begin{array}{c} A_{1}=\left(\begin{array}{cccc} 0 & \alpha & -\beta S & 0\\ 0 & 0 & \nu & \lambda \end{array}\right),\\ A_{2}=\left(\begin{array}{cccc} -\left(\theta +q+b\right) & 0 & \beta S & 0\\ \theta & -\left(\alpha +\eta_{1}+b\right) & 0 & 0\\ \left(1-\omega \right)q & \eta_{1} & -\left(\eta_{2}+\nu +\delta +b\right) & 0\\ \omega q & 0 & \eta_{2} & -\left(\lambda +\delta +b\right) \end{array}\right). \end{array}$$

*A*_2_ represents a Metzler matrix where its diagonal elements are negatives while the off-diagonal elements are nonnegative.

### 3.9. Global Stability of Endemic Equilibrium Point

The stability analysis explains the behavior of epidemic near the equilibrium points. The logarithmic Lyapunov function was proposed by Korobeinikov and Wake [29] to prove the global stability of endemic equilibrium for SIS, SIR, and SIRS models.

**Theorem 8 .**

The endemic equilibrium point *W*^∗^ is asymptotically stable when *R*_0_ > 1 and unstable when *R*_0_ < 1.

**Proof**

The logarithmic Lyapunov function is used to analyze the stability of the endemic equilibrium and is given in the form

(59) $$\begin{array}{c} W=\overset{6}{\underset{i=1}{\sum }}a_{i}\left(X_{i}-x_{i}^{*}\ln\left(X_{i}\right)\right), \end{array}$$

where *a*_*i*_ represents a positive constant, *X*_*i*_ represents some free virus in compartment *i*, and *X*_*i*_^∗^ denotes the number of free viruses in compartment *i* at the equilibrium point. Then, model system (2) is now written as follows:

(60) $$\begin{array}{c} W\left(S,E,Q,I,H,R\right)=\left\{A_{1}\left(S-S^{*}\ln\left(S\right)\right)+A_{2}\left(E-E^{*}\ln\left(E\right)\right)+A_{3}\left(Q-Q^{*}\ln\left(Q\right)\right)+A_{4}\left(I-I^{*}\left.\ln\right]\left(I\right)\right)+A_{5}\left(H-H^{*}\ln\left(H\right)\right)+A_{6}\left(R-R^{*}\ln\left(R\right)\right)\right. \end{array}$$

The constants *A*_1_, *A*_2_, *A*_3_, *A*_4_, *A*_5_, and *A*_6_ are nonnegative constants and the function *W* which is continuous and differentiable. Consider the derivative with respect to each compartment

(61) $$\begin{array}{c} \frac{dW}{dt}=\left\{\begin{array}{c} A_{1}\left(1-\frac{S^{*}}{S}\right)\frac{dS}{dt}+A_{2}\left(1-\frac{E^{*}}{E}\right)\frac{dE}{dt}+A_{3}\left(1-\frac{Q^{*}}{Q}\right)\frac{dQ}{dt}+A_{4}\left(1-\frac{I^{*}}{I}\right)\frac{dI}{dt}\\ +A_{5}\left(1-\frac{H^{*}}{H}\right)\frac{dH}{dt}+A_{6}\left(1-\frac{R^{*}}{R}\right)\frac{dR}{dt}. \end{array}\right.\\ \frac{dW}{dt}=\left\{\begin{array}{c} A_{1}\left(1-\frac{S^{*}}{S}\right)\left(\mu +\alpha Q+\rho R-\beta IS-bS\right)+A_{2}\left(1-\frac{E^{*}}{E}\right)\left(\beta IS-\left(\theta +q+b\right)E\right)\\ +A_{3}\left(1-\frac{Q^{*}}{Q}\right)\left(\phi +\theta E-\left(\alpha +\eta_{1}+b\right)Q\right)\\ +A_{4}\left(1-\frac{I^{*}}{I}\right)\left(\left(1-\omega \right)qE+\eta_{2}I-\left(\eta_{2}+\nu +\delta +b\right)I\right)\\ +A_{5}\left(1-\frac{H^{*}}{H}\right)\left(\omega qE+\eta_{2}I-\left(\lambda +\delta +b\right)H\right)\\ +A_{6}\left(1-\frac{R^{*}}{R}\right)\left(\lambda H+\nu I-\left(\rho +b\right)R\right). \end{array}\right. \end{array}$$

At the endemic equilibrium point,

(62) $$\begin{array}{c} \begin{array}{c} \begin{array}{c} \begin{array}{c} \mu =\beta IS+bS-\alpha Q-\rho R,\\ \beta IS=\left(\theta +q+b\right)E^{*}, \end{array}\\ \phi +\theta E=\left(\alpha +\eta_{1}+b\right)Q^{*},\\ \left(1-\omega \right)qE+\eta_{1}Q=\left(\eta_{1}+\nu +\delta +b\right)I^{*}, \end{array}\\ \omega qE+\eta_{2}I=\left(\lambda +\delta +b\right)H^{*},\\ \lambda H+\nu I=\left(\rho +b\right)R^{*}. \end{array} \end{array}$$

(63) $$\begin{array}{c} \frac{dW}{dt}=\left\{\begin{array}{c} A_{1}\left(\frac{S-S^{*}}{S}\right)\left(bS^{*}-bS\right)+A_{2}\left(\frac{E-E^{*}}{E}\right)\left(\theta +q+b\right)\left(E^{*}-E\right)\\ +A_{3}\left(\frac{Q-Q^{*}}{Q}\right)\left(\alpha +\eta_{1}+b\right)\left(Q^{*}-Q\right)+A_{4}\left(\frac{I-I^{*}}{I}\right)\left(\eta_{1}+\nu +\delta +b\right)\left(I^{*}-I\right)\\ +A_{5}\left(\frac{H-H^{*}}{H}\right)\left(\lambda +\delta +b\right)\left(H^{*}-H\right)+A_{6}\left(\frac{R-R^{*}}{R}\right)\left(\rho +b\right)\left(R^{*}-R\right), \end{array}\right. \end{array}$$

where Equation (63) gives

(64) $$\begin{array}{c} \frac{dW}{dt}=-bA_{1}\frac{{\left(S-S^{*}\right)}^{2}}{S}-\left(\theta +q+b\right)A_{2}\frac{{\left(E-E^{*}\right)}^{2}}{E}-\left(\alpha +\eta_{1}+b\right)A_{3}\frac{{\left(Q-Q^{*}\right)}^{2}}{Q}-\left(\eta_{1}+\nu +\delta +b\right)A_{4}\frac{{\left(I-I^{*}\right)}^{2}}{I}-\left(\lambda +\delta +b\right)A_{5}\frac{{\left(H-H^{*}\right)}^{2}}{H}-\left(\rho +b\right)A_{6}\frac{{\left(R-R^{*}\right)}^{2}}{R}. \end{array}$$

When *S*⟶*S*^∗^, *E*⟶*E*^∗^, *Q*⟶*Q*^∗^, *I*⟶*I*^∗^, *H*⟶*H*^∗^, and *R*⟶*R*^∗^. Therefore, (*dW*/*dt*) ≤ 0 or zero and the function *W* is negative when *W*(*S*, *E*, *Q*, *I*, *H*, *R*) ≥ 0.

By following the approach of [29], the largest invariant set in Δ is a singleton set *W* which is the endemic equilibrium point, and using LaSalle [30] invariant principle, *W*^∗^ is globally asymptotically stable when *R*_0_ > 1 in Δ.

## 4. Numerical Simulation

A series of numerical results for system (2) of the model equations are presented. The explicit Runge-Kutta fourth-order method is considered for solving the first-order ordinary differential equations of *SEQIHR* model numerically with a given initial condition. Partial Rank Correlation Coefficient (PRCC) was used to show the sensitivity analysis of the parameters and basic reproduction number. Parameter values from the literature reviews were used, and some were assumed as shown in Table 3. The data is simulated by substituting them in *R*_0_. The sensitivity index of each partial basic reproduction number *R*_0_ for its parameters.

### 4.1. Sensitivity Analysis and Uncertainty

The sensitivity analysis for the endemic threshold tells us the importance of each parameter for the transmission of COVID-19 disease. The information is crucial for the analysis of complex systems. We used the sensitivity analysis of the parameters to determine the strongness of the *SEQIHR* model predictions for the parameter values. There are usually errors in the data collected and in the initial values assumed for the parameters [35]. The standard equation of a sensitivity index for *R*_0_ is given by

(65) $$\begin{array}{c} \Gamma_{L}^{R_{0}}=\frac{\partial R_{0}}{\partial L}\times \frac{L}{R_{0}}, \end{array}$$

.

From Table 3, it is observed that the *η*_1_ parameter is more sensitive since it increases the basic reproductive number by Γ_*L*_^*R*_0_^ = 1.2813. The increase of this parameter means that in quarantine, people are more stressed such that the immune system decreases in its efficiency, so the virus spreads within the body. The virus causes blood clotting because the virus fights the respiratory system and enters the bloodstream through lung capillaries that are adjacent to the alveolus [36]. The PRCC supported graphically in Figure 2 shows that *η*_1_ has impact on the transmission of COVID-19 disease. *SEQIHR* model shows that hospitalized patients from the infected class are less stressed than those in quarantine, although it also increases the basic reproduction number by (Γ_*L*_^*R*_0_^ = 0.8448); then *η*_1_>*η*_2_. Other sensitive parameters are *θ* with Γ_*L*_^*R*_0_^ = 1.2614, *β* and *μ* which both have Γ_*L*_^*R*_0_^ = 1. Parameters, *ω* and *b*, have the least values which are -0.0717 and -0.9566, respectively, meaning that decreasing *ω* and *b* by a certain percentage always decreases *R*_0_ by the same percentage and the same thing happens if we increase *R*_0_. It shows that if most of the patients are hospitalized, the disease will decrease, and subsequently, there will be no more transmission within the community. Despite the fact that the other parameters have small values, they still increase *R*_0_ by their respective percentages.

From Figure 2, *η*_1_ is positively and highly correlated with *R*_0_ as the absolute value of its PRCC value is higher than the corresponding value of other parameters. Furthermore, natural death *b* is highly negatively correlated with *R*_0_.

#### 4.1.1. Dynamic Population Simulation with a *SEQIHR* Model

The numerical simulation of the *SEQIHR* model variables is shown in Figure 3. We observe that the susceptible class declines to acquire the endemic equilibrium level exponentially as people die naturally or due to the disease. The exposed, quarantined, and infected populations both assume a parabolic curve which increases exponentially to a certain maximum point before they decelerate to an endemic level. Hospitalized and recovered populations both assumed a parabolic shape as it increases exponentially to a certain maximum point before decelerating to an endemic point.

#### 4.1.2. Relationship between Most Positive and Negative Parameters with Basic Reproduction Number *R*_0_

From Section 4.1, we observed that the most positive parameter is *η*_1_. The relationship between *η*_1_ and *R*_0_ is shown in Figure 4(a), whereby we noticed that the increase of stress results in a quick rise of *R*_0_. This shows that individuals isolated from their families are more stressed, which increases the disease infection because stress lowers body immunity. Similarly, the natural death *b* is the most negative sensitive parameter shown in Figure 4(b), which means that any reduction in it will make the basic reproduction number experience significant exponential retardation.

#### 4.1.3. Simulation of Stability Analysis of *SEQIHR* Model

The numerical simulations for the stability analysis are performed to the analytical results of the model. For the equilibrium point to be globally asymptomatic stable, the model trajectories for the state variables should be originated from different initial values and sometimes converge to a common point and maintain an endemic equilibrium point. But if the model trajectories for state variables remain near the equilibrium point and move together in the long run, this implies that the equilibrium point is globally stable. The six trajectories in each class are represented by different colors as shown by a legend that converge towards equilibrium point as time approaches infinity. The model variables *S*, *E*, *Q*, *I*, *H*, and *R* varied by considering Figures 5(a) and 7(b), respectively, are illustrated as follows:

#### 4.1.4. Control Parameters

By considering the variation of some control parameters; from Figure 8(a), when the contact rate (*β*) increases, the decaying population rate also increases, but when the contact rate decreases, the decaying rate also decreases. From Figure 8(b), when the contact rate increases, the infections also increase and apply the same when the contact rate decreases and the infections decreases. When stress increases in the susceptible class, the rate of decaying increases, and if the stress decreases, the decaying rate decreases, as shown in Figure 9(a). From Figure 9(b), when stress (*η*_1_) increases, the rate of infection increases, and when *η*_1_ decreases, then the rate of infected population decreases. Moreover, when *η*_2_ increases, the rate of infected and hospitalized increases and then decreases when *η*_2_ decreases as in Figures 10(a) and 10(b).

#### 4.1.5. Parameter Identifiability and Model Fitting

The identifiability of parameters is essential to the proposed *SEQIHR* model. Such parameters are *β*, *μ*, *ω*, *α*, *η*_1_, and *η*_2_. Parameter identifiability is implemented by using the least square method to minimize the sum of squared differences between the observations and the *SEQIHR* model [37] and is defined as

(66) $$\begin{array}{c} SS\left(\theta \right)=\overset{n}{\underset{i=1}{\sum }}{\left[y_{i}-f\left(x_{i},\theta \right)\right]}^{2}, \end{array}$$

where *y*_*i*_ are the observed data of all compartments, *i* is the number of compartments (i.e., *i* = 1, 2, ⋯, *n*), and *f*(*x*_*i*_, *θ*) is the solution for all compartments of the *SEQIHR* model. With the initial values of the parameters given as *β*, *μ*, *ω*, *α*, *η*_1_, and *η*_2_, the least squares identifiabilities are obtained as shown in Table 4 as the initial value and estimated values and used to fit the simulated data as shown in Figure 11. The relationship of initial parameter values and the identifiable values from the least square method is very close.

## 5. Conclusion

COVID-19 pandemic spread rapidly all over the world, which led to the severe human and socioeconomic burden worldwide. In this study, a mathematical model was developed for the transmission of COVID-19 when a human is stressed. The model consists of six compartments: Susceptible (*S*), Exposed (*E*), Quarantined (*Q*), Infectious (*I*), Hospitalized (*H*), and Recovered (*R*) human population. Initially, the model was formulated and some mathematical analyses were presented, including positivity, invariant region, existence, uniqueness of the solution, and stability results for the disease-free equilibrium. The disease-free equilibrium for both local and global is stable when *R*_0_ < 1 was proved. This exploration suggests that the COVID-19 disease can enter and spread to the human population if *R*_0_ > 1 provided that the initial human population is close to the infested region. But also, die out when few initial human populations are infected and *R*_0_ < 1. The basic reproduction number obtained from this study was 2.1692, which shows that the disease is endemic and unique. The most sensitivity indices are summarized in Table 3, and the least positively and negatively sensitive parameters are crucial for the transmission of COVID-19.

The numerical results in this study showed that stress affects many quarantined people whereby their immune system is disturbed by the COVID-19, and this is most likely because during quarantine, people are isolated from their families and community members, so they develop fear, and later, the body becomes stressed which affects their immune system. When the immune system is disturbed, it fails to fight against the intruders, which leads to the fast spread of COVID-19 throughout the body. Our graphical presentation illustrated that the control parameters showed a great success on minimizing the spread of COVID-19 in the community.

The plan for a future work is to use more detailed and authentic data when having access to COVID-19 data which will be employed in the *SEQIHR* model. Furthermore, we intend to add a vaccination in our model compartment to implement optimal control strategies and extend to a stochastic model. The limitations of this work are the assumption on an equal death in all compartment while in real situation the infected population has a higher death rate than the susceptible population.

## Figures and Tables

**Figure 1:** Schematic flow diagram showing dynamics of COVID-19.

**Figure 2:** Global sensitivity analysis and PRCC results for *R*_0_.

**Figure 3:** Dynamic simulation of a *SEQIHR* model.

**Figure 4:** Effect of stress *η*_1_ and natural death *b* on *R*_0_.

**Figure 5:** Global stability of endemic equilibrium for susceptible and exposed human population.

**Figure 6:** Global stability of endemic equilibrium for quarantined and infected human population.

**Figure 7:** Global stability of endemic equilibrium for hospitalized and recovered human population.

**Figure 8:** Variation of contact rate *β* in susceptible and infected population.

**Figure 9:** Variation of *η*_1_ in susceptible and infected human population.

**Figure 10:** Variation of *η*_2_ in infected and hospitalized human population.

**Figure 11:** Fitted graphs.

**Table 1:** Model variable description.

Variables	Description
*S*(*t*)	Number of susceptible population at time *t*
*Q*(*t*)	Number of quarantined population at time *t*
*E*(*t*)	Number of exposed population at time *t*
*I*(*t*)	Number of infectious population at time *t*
*H*(*t*)	Number of hospitalized population at time *t*
*R*(*t*)	Number of recovered population at time *t*

**Table 2:** Model parameter description.

Parameters	Description
*β*	Contact rate (effective transmission rate)
*μ*	Recruitment rate to the susceptible population
*b*	Human natural death rate
*ϕ*	Quarantined population from infected countries
*ρ*	Recovered population rate back to susceptible class
*α*	Population rate after the quarantined period to susceptible
*ν*	Recovery rate from infected population
*λ*	Recovered rate from hospitalized population
*ω*	Proportion of exposed population with contradicting symptoms
*q*	Progression rate from exposed to hospitalized and infectious classes
*θ*	Proportion of exposed population with no symptoms
*η*_1_	Stress to the infected population from quarantine
*η*_2_	Stress to the hospitalized population from infectious class
*δ*	Death due to the disease from infectious and hospitalized classes

**Table 3:** Parameter values and sensitivity indices.

Parameter	Values	Sources	Sensitivity index value
*β*	0.015	Assumed	1.0000
*μ*	8.94	Assumed	1.0000
*ω*	0.083	Assumed	-0.0388
*b*	0.0104	[31]	-0.9483
*α*	0.85	Assumed	0.7100
*ν*	0.07	[32]	0.090
*θ*	0.2435	[33]	1.2614
*η*_1_	0.85	Assumed	1.2813
*η*_2_	0.65	Assumed	0.8448
*δ*	0.039	[34]	0.0507
*q*	0.099	Assumed	0.7092

**Table 4:** Parameter identifiability.

Parameter	Initial values	Estimated values
*β*	0.015	0.0147
*μ*	8.94	9.8
*ω*	0.083	0.096
*b*	0.0104	0.013
*α*	0.85	1.1
*ν*	0.07	0.063
*θ*	0.2435	0.224
*η*_1_	0.85	0.72
*η*_2_	0.65	0.51
*δ*	0.039	0.038
*q*	0.099	0.098
*ρ*	0.003	0.0032
*λ*	0.002	0.0018
*ϕ*	0.001	0.0009

## Data Availability

Some data used in our numerical simulation (as shown in Table 3) are assumed and others from published articles as cited in this work.
